This article has been retracted.

# MABAC method for multiple attribute group decision making under single-valued neutrosophic sets and applications to performance evaluation of sustainable microfinance groups lending

**DOI:** 10.1371/journal.pone.0280239

**Published:** 2023-01-11

**Authors:** Hui Ran

**Affiliations:** College of Finance and Logistics Management, LiuZhou Vocational & Technical College, Liuzhou, 545006, Guangxi, China; Hefei University of Technology, CHINA

## Abstract

As an important supplement to my country’s financial institutions, micro-loan companies serve "agriculture, rural areas and farmers", small and micro enterprises, and individuals, to a certain extent, alleviating the financing difficulties of such groups and regulating private finance. However, micro-loan companies only lend but do not deposit. In the process of lending, due to inadequate risk management, the risk problem has become increasingly prominent. With the continuous growth of the loan amount of rural credit and the continuous increase of microfinance groups lending customers, it faces certain problems in its risk management, which increases the risks of the company in all aspects. The performance evaluation of sustainable microfinance groups lending is a classical MAGDM issues. In such paper, the Hamming distances of single-valued neutrosophic sets (SVNSs) and maximizing deviation method (MDM) is used to obtain the attribute weights and the single-valued neutrosophic numbers MABAC(SVNN-MABAC) method is structured for MAGDM under SVNSs. Finally, an example about performance evaluation of sustainable microfinance groups lending and some comparative decision analysis are given to proof the SVNN-MABAC.

## 1. Introduction

The MADM is a kind of very complex optimization decision-making problem, which often occurs in the field of decision engineering, economics, military, and public management [1–5]. In the process of MADM, the value of decision-making attributes often has information uncertainty, and the data is difficult to estimate, predict, and evaluate [6–13]. This is more general than the decision attribute value is accurate data and clear information. Decision problems have multiple decision attributes [14–17]. For qualitative decision attributes, the decision attribute values are usually presented in the form of language evaluation, such as excellent, good, qualified, unqualified and other semantic information, which brings difficulties to mathematical calculation and analysis, simply quantitative conversion of semantic information, such as setting grades, cannot guarantee scientificity, and it is easy to lose important information, resulting in decision-making mistakes [18–22]. Zadeh [23] structured the fuzzy sets (FSs). Then, Atanassov [24] structured defined intuitionistic fuzzy sets (IFSs). Liu et al. [25] defined the Dombi BM operations for MAGDM. Smarandache [26] structured the neutrosophic sets (NSs). However, considering that the medium intelligence set is defined in a non-standard sub interval, which is not convenient for application in engineering and natural science, Wang et al. [27] proposed the SVNSs to solve this problem. It is a subclass of the medium intelligence set. It uses true membership, false membership and uncertainty functions to describe decision information together, which can be easily applied in engineering, science and other fields. SVNSs have many obvious advantages in dealing with uncertain and fuzzy decision information, and a lot of research has been done on this. Biswas, Pramanik and Giri [28] used SVNSs to represent decision information and TOPSIS to propose MADM method. Jiang and Shou [29] proposed the similarity measurement for SVNSs based on Dempster Shafer distance theory. Ye [30] proposed a decision weighted correlation coefficient of SVNSs, and proposed a MADM with cross entropy of SVNSs. The key roles of TOPSIS [31] is that the distance between the optimal scheme and the positive ideal scheme should be the shortest, and the distance between the optimal scheme and the negative ideal scheme should be the farthest. The combination of TOPSIS method [32–37] and SVNSs [38–49] can effectively solve the MADM problem [50–59].

There are three shortcomings in disposing of the MAGDM problems under SVNNs environment that to form our incentives in the following:

(1) The existing decision methods have complex computation degree [38–49]. How to investigate the decision methods consider the relatively simpler computation degree is an interesting and hot topic. For this reason, the first incentive of this paper is to build the new relatively simpler decision methods.

(2) The existing weight methods just consider completely known weight information [32–37]. How to investigate the weight consider completely unknown weight is an interesting and hot topic. For this reason, the second incentive of this paper is to design the new weight method, which can deal with completely unknown weight.

(3) The timely innovation of group lending technology of microfinance is important for promoting the innovation of financial support for agricultural products in the implementation of China’s rural revitalization strategy [60–65]. It is of practical value and theoretical significance to promote the innovation of financial support for agricultural products in the implementation of China’s rural revitalization strategy and to bridge the theoretical controversy of microcredit loan technology. The performance evaluation of sustainable microfinance groups lending in Chinese is still in a blank state. Therefore, it is urgent for researchers in related disciplines to conduct exploratory research in this field to enrich the research content of performance evaluation of sustainable microfinance groups lending in my country. The performance evaluation of sustainable microfinance groups lending is a classical MAGDM issues. Thus, the third incentive of this paper is to build new decision methods for performance evaluation of sustainable microfinance groups lending.

On this basis, combined with the characteristics of performance evaluation of sustainable microfinance groups lending, a new MAGDM method for performance evaluation of sustainable microfinance groups lending in SVNNs environment is proposed. Specific research points are listed as follows:

(1) In this paper, the SVNN-MABAC method is built based on the MABAC [66] and SVNNs with completely unknown weight information. The SVNN-MABAC investigate the decision methods consider the distances-based measures degree.

(2) For deriving the completely known weight of the attribute, an optimization model is built on the MDM method, by which the attribute weights can be decided. Then, the optimal alternative is chosen through calculating the maximizing deviation among different alternatives. Then, combine the traditional MABAC model with SVNNs information, the SVNN-MABAC method is established and the computing steps for MAGDM are built.

(3) The main advantages of the SVNN-MABAC method are given as follows: the computing results by SVNN-MABAC method are stable; the calculating equations are simple; it takes the latent values of gains and losses into account; it is available to combine this model with other approaches. Hence, the SVNN-MABAC method is a good tool to derive reasonable decision-making results.

(4) Finally, a numerical example for performance evaluation of sustainable microfinance groups lending has been given and some comparisons is used to illustrate advantages of SVNN-MABAC. This paper mainly provides method guidance and technical support for the realization of SVNN-MABAC. This has far-reaching significance for the decision-making of sustainable microfinance groups lending in the public sector, infrastructure construction and even national security and stability.

In order to do, the reminder of our paper proceeds. The SVNSs is reviewed in Sec. 2. The SVNN-MABAC method for MAGDM is defined in Sec. 3. An example for performance evaluation of sustainable microfinance groups lending is given to show the superiority in Sec. 4. the conclusion is fully given in Sec. 5.

## 2. Preliminaries

Wang et al. [27] defined the given SVNSs

**Definition 1** [27]. The SVNSs *A* in *Y* is defined:

YA={(y,AT(y),AI(y),AF(y))|y∈Y} (1)

with defined truth-membership *AT*(*y*), defined indeterminacy-membership *AI*(*y*) and defined falsity-membership *AF*(*y*), *AT*(*y*), *AI*(*y*), *AF*(*y*)∈[0,1], 0≤*ATy*+*AI*(*y*)+*AF*(*y*)≤3.

The SVNN is expressed as *YA* = (*AT*,*AI*,*AF*), *AT*,*AI*,*AF*∈[0,1], 0≤*AT*+*AI*+*AF*≤3.

**Definition 2 [67]**. Let *YA* = (*AT*,*AI*,*AF*) be the SVNN, the score value is:

$$SV(YA)=\frac{\left(2+AT-AI-AF\right)}{3},\;SV(YA)\in [0,1].$$ (2)

**Definition 3 [67].** Let *YA* = (*AT*,*AI*,*AF*) be the SVNN, the accuracy value is:

HV(YA)=AT−AF,HV(YA)∈[−1,1] (3)

Peng et al.[67] came up with order decision relation for SVNNs.

**Definition 4 [67].** Let *YA* = (*AT*,*AI*,*AF*) and *YB* = (*BT*,*BI*,*BF*) be two given SVNNs, let $SV(YA)=\frac{\left(2+AT-AI-AF\right)}{3}$ and $SV(YB)=\frac{\left(2+BT-BI-BF\right)}{3}$, and let *HV*(*YA*) = *AT*−*AF* and *HV*(*YB*) = *BT*_*B*_−*BF*, if *SV*(*YA*)<*SV*(*YB*), *YA*<*YB*; if *SV*(*YA*) = *SV*(*YB*), then (1)if *HV*(*YA*) = *HV*(*YB*), *YA* = *YB*; (2) if *HV*(*YA*)<*HV*(*YB*), *YA*<*YB*.

**Definition 5 [68].** Let *YA* = (*AT*,*AI*,*AF*) and *YB* = (*BT*,*BI*,*BF*) be two SVNNs, the basic operations are defined:

$$\begin{array}{l} (1)\;YA⊕YB=(AT+BT-AT\cdot BT,AI\cdot BI,AF\cdot BF);\\ (2)\;YA⊗YB=(AT\cdot BT,AI+BI-AI\cdot BI,AF+BF-AF\cdot BF);\\ (3)\;\lambda YA=(1-{\left(1-AT\right)}^{\lambda },{\left(AI\right)}^{\lambda },{\left(AF\right)}^{\lambda }),\lambda >0;\\ (4)\;{\left(YA\right)}^{\lambda }=({\left(AT\right)}^{\lambda },{\left(AI\right)}^{\lambda },1-{\left(1-AF\right)}^{\lambda }),\lambda >0. \end{array}$$

**Definition 6 [69].** Let *YA* = (*AT*,*AI*,*AF*) and *YB* = (*BT*,*BI*,*BF*), then the Hamming distance between *YA* = (*AT*,*AI*,*AF*) and *YB* = (*BT*,*BI*,*BF*) is defined:

$$HD(YA,YB)=\frac{\left|AT-BT|+|AI-BI|+|AF-BF\right|}{3}$$ (4)

## 3. The MABAC method for MAGDM with SVNNs

Let *ZZ* = {*ZZ*_1_,*ZZ*_2_,…,*ZZ*_*n*_} be the set of attributes, *wz* = {*wz*_1_,*wz*_2_,…*wz*_*n*_} be the weight of attributes *ZZ*_*j*_. Let *PP* = {*PP*_1_,*PP*_2_,…,*PP*_*m*_} be alternatives. And *AQ* = (*qq*_*ij*_)_*m*×*n*_ = (*AT*_*ij*_,*AI*_*ij*_,*AF*_*ij*_)_*m*×*n*_ is the SVNN matrix. Integrating the MABAC method for MAGDM with SVNNs, we build the SVNN-MABAC method with SVNNs. The SVNN-MABAC procedures can be described subsequently.

**Step 1.** Set up the SVNN matrix *AQ* = (*aq*_*ij*_)_*m*×*n*_ = (*AT*_*ij*_,*AI*_*ij*_,*AF*_*ij*_)_*m*×*n*_.


$$AQ={\left(aq_{ij}^{}\right)}_{m\times n}=[\begin{array}{cccc} aq_{11} & aq_{12} & \ldots & aq_{1n}\\ aq_{21} & aq_{22} & \ldots & aq_{2n}\\ \vdots & \vdots & \vdots & \vdots \\ aq_{m1} & aq_{m2} & \ldots & aq_{mn} \end{array}]$$ (5)

**Step 2.** Normalize matrix *AQ* = (*qq*_*ij*_)_*m*×*n*_ to *NQ* = [*nq*_*ij*_]_*m*×*n*_.


$$\begin{array}{l} nq_{ij}=(NT_{ij},NI_{ij},NF_{ij})\\ =\left\{ \begin{array}{c} (AT_{ij},AI_{ij},AF_{ij}),\;ZZ_{j}\;is\;a\;benefit\;criterion\\ (AF_{ij},AI_{ij},AT_{ij}),\;ZZ_{j}\;is\;a\;\mathrm{cost}\;criterion \end{array}\right. \end{array}$$ (6)

**Step 3.** Utilize the MDM to determine the weight of attributes.

The MDM [70] is used to derive the weight values.

**(1)** Depending on the *NQ* = [*nq*_*ij*_]_*m*×*n*_, the deviation of *PP*_*i*_ from other alternatives is calculated.

$$SVNNHD_{ij}=\sum_{t=1}^{m}wz_{j}\cdot HD(nq_{ij},nq_{ij})$$ (7)

where $HD(nq_{{}_{ij}},nq_{ij})=\frac{\left|NT_{ij}-NT_{tj}|+|NI_{ij}-NI_{tj}|+|NF_{ij}-NF_{tj}\right|}{3}$.

**(2)** Calculate the weighted deviation.


$$\begin{array}{l} SVNNHD_{j}(wz)=\sum_{i=1}^{m}SVNNHD_{ij}(wz)\\ =\sum_{i=1}^{m}\sum_{t=1}^{m}wz_{j}\left(\frac{\left|NT_{ij}-NT_{tj}|+|NI_{ij}-NI_{tj}|+|NF_{ij}-NF_{tj}\right|}{3}\right) \end{array}$$ (8)

**(3)** Construct the programming model.


$$\left(M-1)\{\begin{array}{l} \max D(wz)=\sum_{j=1}^{n}\sum_{i=1}^{m}\sum_{t=1}^{m}wz_{j}(\frac{\left|NT_{ij}-NT_{tj}|+|NI_{ij}-NI_{tj}|+|NF_{ij}-NF_{tj}\right|}{3})\\ s.t.\;{\mathrm{wz}}_{j}\geq 0,\;\sum_{j=1}^{n}wz_{j}^{2}=1 \end{array}\right)$$ (9)

To solve this defined model, The Lagrange function is used to solve this model.

$$L(wz,\xi )=\sum_{j=1}^{n}\sum_{i=1}^{m}\sum_{t=1}^{m}wz_{j}(\frac{\left|NT_{ij}-NT_{tj}|+|NI_{ij}-NI_{tj}|+|NF_{ij}-NF_{tj}\right|}{3})+\frac{\xi }{2}(\sum_{j=1}^{n}wz_{j}^{2}-1)$$

where *ξ* is the Lagrange decision multiplier, the partial derivatives are obtained.


$$\left\{ \begin{array}{l} \frac{\partial L}{\partial wz_{j}}=\sum_{i=1}^{m}\sum_{t=1}^{m}(\frac{\left|NT_{ij}-NT_{tj}|+|NI_{ij}-NI_{tj}|+|NF_{ij}-NF_{tj}\right|}{3})+\xi wz_{j}=0\\ \frac{\partial L}{\partial \xi }=\frac{1}{2}\left(\sum_{j=1}^{n}wz_{j}^{2}-1\right)=0 \end{array}\right.$$

And the weight information is obtained.


$$wz_{j}^{*}=\frac{\sum_{i=1}^{m}\sum_{t=1}^{m}\left|NT_{ij}-NT_{tj}|+|NI_{ij}-NI_{tj}|+|NF_{ij}-NF_{tj}\right|}{\sqrt{\sum_{j=1}^{n}{\left(\sum_{i=1}^{m}\sum_{t=1}^{m}\left(\left|NT_{ij}-NT_{tj}|+|NI_{ij}-NI_{tj}|+|NF_{ij}-NF_{tj}\right|\right)\right)}^{2}}}$$

Finally, the normalized weights are obtained.


$$wz_{j}=\frac{\sum_{i=1}^{m}\sum_{t=1}^{m}\left(\left|NT_{ij}-NT_{tj}|+|NI_{ij}-NI_{tj}|+|NF_{ij}-NF_{tj}\right|\right)}{\sum_{j=1}^{n}\sum_{i=1}^{m}\sum_{t=1}^{m}\left(\left|NT_{ij}-NT_{tj}|+|NI_{ij}-NI_{tj}|+|NF_{ij}-NF_{tj}\right|\right)}$$ (10)

**Step 4.** Obtain the weighted matrix *OQ* = (*oq*_*ij*_)_*m*×*n*_:

$$\begin{array}{l} oq_{ij}=(WNT_{ij},WNI_{ij},WNF_{ij})\\ =wz_{j}\cdot nq_{ij}=\left(1-{\left(1-NT_{ij}\right)}^{wz_{j}},{\left(NI_{ij}\right)}^{wz_{j}},{\left(NF_{ij}\right)}^{wz_{j}}\right) \end{array}$$ (11)

**Step 5.** Obtain the defined SVNN border approximation area (SVNNBAA) *GQ* = (*gq*_*j*_)_1×*n*_.


gqj=∏i=1m(oqij)1m=(∏i=1m(WNTij)1m,∏i=1m(WNIij)1m,1−∏i=1m(1−WNFij)1m) (12)

**Step 6.** Obtain the SVNN distance decision matrix *DQ* = (*dq*_*ij*_)_*m*×*n*_ from SVNNBAA with Eq (13).


$$dq_{ij}=\{\begin{array}{l} (HD(oq_{ij},gq_{j})),\;if\;SV(oq_{ij})\geq S(gq_{j}),\\ -HD(oq_{ij},gq_{j}),\;if\;SV(oq_{ij})<S({\mathrm{gq}}_{j}), \end{array}$$ (13)

**Step 7.** Obtain the final order value *SVNNF*_*i*_.


$$SVNNF_{i}=\sum_{j=1}^{n}dq_{ij}$$ (14)

**Step 8.** The given alternatives can be order with *SVNNF*_*i*_. The higher information value of *SVNNF*_*i*_ is, the optimal selection will be.

## 4. The empirical example and comparative analysis

### 4.1 An empirical example

Microfinance is an institutionalized form of credit that provides credit services to the low-income poor. Starting from the mid-1970s, some developing countries in Asia and Latin America, recognizing the disadvantaged position of the poor in the formal financial market, borrowed some features of traditional private credit and modern management experience, combined with the economic and social conditions of the countries where they are located and the economic and cultural characteristics of the poor, and on the basis of continuous exploration and experimentation, creatively constructed a variety of Credit systems and methods. Since most of the institutional arrangements of such credit modalities are aimed at the self-employed poor with normal production capacity, and they are designed to treat the self-employed poor households and the economic activities they are engaged in as micro-enterprises. Under these assumptions, this type of credit service for the poor is referred to as microenterprise credit or microcredit for short. When this approach was introduced in our country, it was translated as microcredit. The situation between Internet financial enterprises and traditional commercial banks is not a "zero-sum game". Compared with traditional financial service products, Internet financial wealth management products are more substitutable. In this context, subject to the gradually approaching market pressure of Internet finance, traditional commercial banks must actively carry out reforms and innovations if they want to calmly deal with and reverse the adversity. Therefore, commercial banks must change the traditional commercial banking business operation model of "sugar daddy, large households, relying on resources, and profit margins", and actively take measures to deal with the crises and challenges brought by Internet financial products. In recent years, the development momentum of my country’s Internet finance has been particularly rapid. However, with the continuous decision improvement of the socialist market economic with Chinese characteristics, the industry environment for the development of my country’s Internet finance has been gradually standardized, but at the same time, new problems have emerged. From the perspective of the development of microfinance business, Internet finance has spawned a wide variety of business products. However, due to the influence of factors such as lack of industry supervision, commercial banks’ microfinance business risk events frequently occur, which is not conducive to commercial banks’ sustainable operations. The performance evaluation of sustainable microfinance groups lending is the MAGDM. In this paper, an empirical application of performance evaluation of sustainable microfinance groups lending will be provided with SVNN-MABAC. There are five microfinance groups *PP*_*i*_(*i* =1,2,3,4,5) are to evaluated the performance of sustainable microfinance groups lending. In order to assess these microfinance groups fairly, the experts group give their assessment with four defined attributes: ①ZZ_1_ is the pay back ability; ②ZZ_2_ is the loan amount; ③ZZ_3_ is the loan utilization rate; ④ZZ_4_ is the loan repayment ability. Evidently, ZZ_2_ is the cost, others are the benefit. Then, the SVNN-MABAC method is applied to MAGDM for solving the performance evaluation of sustainable microfinance groups lending with SVNNs. The built SVNN-MABAC method involves the following steps:

**Step 1.** Set up the SVNN-matrix *AQ* = (*aq*_*ij*_)_5×4_ as in Table 1.

**Table 1:** SVNN information.

	ZZ_1_	ZZ_2_	ZZ_3_	ZZ_4_
PP_1_	(0.53, 0.35, 0.37)	(0.26, 0.25, 0.22)	(0.50, 0.35, 0.50)	(0.33, 0.33, 0.35)
PP_2_	(0.55, 0.25, 0.55)	(0.58, 0.53, 0.23)	(0.52, 0.07, 0.59)	(0.55, 0.23, 0.55)
PP_3_	(0.35, 0.07, 0.55)	(0.53, 0.32, 0.38)	(0.53, 0.07, 0.58)	(0.53, 0.29, 0.58)
PP_4_	(0.33, 0.33, 0.33)	(0.52, 0.02, 0.22)	(0.55, 0.53, 0.55)	(0.33, 0.33, 0.36)
PP_5_	(0.35, 0.09, 0.35)	(0.32, 0.05, 0.29)	(0.59, 0.35, 0.53)	(0.33, 0.33, 0.33)

**Step 2.** Normalize *AQ* = (*aq*_*ij*_)_5×4_ to *NQ* = [*nq*_*ij*_]_5×4_ (See Table 2).

**Table 2:** The normalized SVNN information.

	ZZ_1_	ZZ_2_	ZZ_3_	ZZ_4_
PP_1_	(0.53, 0.35, 0.37)	(0.22, 0.25, 0.26)	(0.50, 0.35, 0.50)	(0.33, 0.33, 0.35)
PP_2_	(0.55, 0.25, 0.55)	(0.23, 0.53, 0.58)	(0.52, 0.07, 0.59)	(0.55, 0.23, 0.55)
PP_3_	(0.35, 0.07, 0.55)	(0.38, 0.32, 0.53)	(0.53, 0.07, 0.58)	(0.53, 0.29, 0.58)
PP_4_	(0.33, 0.33, 0.33)	(0.22, 0.02, 0.52)	(0.55, 0.53, 0.55)	(0.33, 0.33, 0.36)
PP_5_	(0.35, 0.09, 0.35)	(0.29, 0.05, 0.32)	(0.59, 0.35, 0.53)	(0.33, 0.33, 0.33)

**Step 3.** Obtain the attribute weights in Table 3.

**Table 3:** The attributes weights.

	ZZ_1_	ZZ_2_	ZZ_3_	ZZ_4_
*wz*_*j*_	0.2574	0.1898	0.2667	0.2861

**Step 4.** Obtain the weighted matrix *OQ* = (*oq*_*ij*_)_*m*×*n*_ (Table 4).

**Table 4:** SVNN weighted normalized values.

ZZ_1_	ZZ_2_
(0.2266, 0.2078, 0.2624)	(0.2066, 0.2427, 0.2642)
(0.2262, 0.2406, 0.4626)	(0.4404, 0.2246, 0.2468)
(0.2242, 0.4224, 0.4644)	(0.4026, 0.2422, 0.4682)
(0.4602, 0.2268, 0.2066)	(0.2400, 0.2422, 0.6200)
(0.2422, 0.4268, 0.2462)	(0.2264, 0.4206, 0.2606)
ZZ_3_	ZZ_4_
(0.4622, 0.4266, 0.4084)	(0.4664, 0.2487, 0.2222)
(0.2244, 0.4264, 0.4442)	(0.2424, 0.2267, 0.4468)
(0.2622, 0.002, 0.2422)	(0.2624, 0.2442, 0.2426)
(0.2226, 0.2008, 0.2622)	(0.2224, 0.28607, 0.2266)
(0.2242, 0.4244, 0.4666)	(0.2020, 0.2067, 0.4660)

**Step 5.** Determine the SVNNBAA (Table 5).

**Table 5:** SVNNBAA.

	SVNNBAA
ZZ_1_	(0.3322, 0.2362, 0.2223)
ZZ_2_	(0.3633, 0.003, 0.3233)
ZZ_3_	(0.3336, 0.3006, 0.3633)
ZZ_4_	(0.2633, 0.2366, 0.2062)

**Step 6.** Calculate the *DQ* = (*dq*_*ij*_)_5×4_ (Table 6).

**Table 6:** Distance matrix.

	ZZ_1_	ZZ_2_	ZZ_3_	ZZ_4_
PP_1_	-0.0837	0.0255	0.0400	-0.1022
PP_2_	0.1320	-0.0690	0.1297	-0.1421
PP_3_	-0.1054	-0.0461	-0.1078	-0.1162
PP_4_	-0.0480	-0.0387	-0.0293	-0.1063
PP_5_	-0.1227	-0.0648	-0.1418	-0.2150

**Step 7.** Calculate *SVNNF*_*i*_ in Table 7.

**Table 7:** The SVNNF values.

Alternative	SVNNF value
PP_1_	-0.1204
PP_2_	0.0506
PP_3_	-0.3755
PP_4_	-0.2223
PP_5_	-0.5443

**Step 8.** From the Table 6, the order is: *PP*_2_>*PP*_1_>*PP*_4_>*PP*_3_>*PP*_5_ and *PP*_2_ is the optimal selection.

### 4.2 Compare analysis

The SVNN-MABAC is made comparison with SVNNWA & SVNNWG operators **[67]**, SVNN-CODAS method [71] and SVNN-EDAS method [72]. The decision results of different methods are in Table 8.

**Table 8:** Results for different given methods.

Methods	Order	The optimal choice	The worst choice
SVNNWA [67]	*PP*_2_>*PP*_4_>*PP*_5_>*PP*_1_>*PP*_3_	*PP*_2_	*PP*_3_
SVNNWG [67]	*PP*_2_>*PP*_4_>*PP*_1_>*PP*_5_>*PP*_3_	*PP*_2_	*PP*_3_
SVNN-CODAS [71]	*PP*_2_>*PP*_1_>*PP*_4_>*PP*_5_>*PP*_3_	*PP*_2_	*PP*_3_
SVNN-EDAS [72]	*PP*_2_>*PP*_5_>*PP*_4_>*PP*_1_>*PP*_3_	*PP*_2_	*PP*_3_
SVNN-MABAC method	*PP*_2_>*PP*_1_>*PP*_4_>*PP*_3_>*PP*_5_	*PP*_2_	*PP*_3_

From Table 8, obviously, the best enterprise given is *PP*_2_ in the five given methods, and the worst selection is *PP*_3_ in most cases. In other words, the order of these five methods have light difference. Different decision methods may effectively solve the MAGDM problem from different research decision angles. These five given models have their given advantages: (1) the SVNNWA operator emphasis group decision influences; (2) the SVNNWG operator emphasis individual decision influences; (3) In the SVNN-CODAS method, the overall performance of the alternatives is measured by Euclidean distance and Hamming distance of negative ideal points, where Euclidean distance is used as the main measure for evaluation. If the Euclidean distance between two alternatives is very close, then the Hamming distance is used to compare the two alternatives. Among them, the closeness of the Euclidean distance can be determined by using the threshold parameter; (4) The SVNN-EDAS method has required fewer computations, although it results in the same ranking of alternatives. The evaluations of alternatives in EDAS method based on distance measures from the average solutions in terms of each criterion unlike TOPSIS and VIKOR. (5) The SVNN-MABAC method has a large amount of precious characteristic, such as: the computing results by SVNN-MABAC method are stable; the calculating equations are simple; it takes the latent values of gains and losses into account; it is available to combine this model with other approaches. Hence, the SVNN-MABAC method is a good tool to derive reasonable decision making results.

## 5. Conclusion

In recent years, the development of Internet finance has shown an unprecedented prosperous trend, which is the result of the rapid decision development of Internet information technology and cloud technology. Under this background, there are endless cases of innovation and entrepreneurship in the domestic Internet finance field, especially the development of Internet wealth management products. Especially quickly. In 2014, Alibaba Finance launched the "Yue Bao" service for the first time, mainly providing Alipay wealth management services. This product is a wealth management fund product jointly launched by Alipay and Tianhong Fund. Money market financial instruments with high security and stability, such as certificates of deposit. Once the Yu’e Bao product was launched, it aroused strong reactions in the financial investment market. It is known as a "wealth management artifact" due to its low threshold and fast receipt of income. Under this wave, other Internet financial companies have followed closely and launched various wealth management products, such as Baidu’s "Baifa", Suning’s "Change Money", Tencent’s "Wealth Management", etc. Financial markets are showing unprecedented prosperity. The performance evaluation of sustainable microfinance groups lending is the MAGDM. In this given paper, the MABAC method is built for SVNN-MAGDM. First, the Hamming distances of SVNSs and MDM is employed to obtained the decision weights and the SVNN-MABAC method is structured for MAGDM under SVNSs. Finally, an example about performance evaluation of sustainable microfinance groups lending and some comparative decision analysis are given to proof the SVNN-MABAC. The main contributions of this work are (1) The attribute weights are obtained by MDM method; (2) the paper constructs the SVNN-MABAC method for performance evaluation of sustainable microfinance groups lending; (3) the established method is illustrated by a case study for performance evaluation of sustainable microfinance groups lending; and (4) some comparisons prove the rationality and advantages.

According to the current research status in this field, research of evaluation methods will be continued in the following aspects in the future. (1) Consensus and consistency improvement should be investigated in group decision-making [73–79] for performance evaluation of sustainable microfinance groups lending. (2) The methods proposed in this paper is improved to consider the expression of evaluation information based on SVNSs, such as group decision method based on probabilistic linguistic information [80,81]and probabilistic uncertain linguistic information [82,83], which is also a topic worthy of future research.
